# Oxidative Stress and Ginsenosides: An Update on the Molecular Mechanisms

**DOI:** 10.1155/2022/9299574

**Published:** 2022-04-20

**Authors:** Bo He, Deyun Chen, Xiaochao Zhang, Renhua Yang, Yuan Yang, Peng Chen, Zhiqiang Shen

**Affiliations:** ^1^School of Pharmaceutical Science & Yunnan Key Laboratory of Pharmacology for Natural Products, Kunming Medical University, Kunming 650500, China; ^2^College of Food, Drugs, and Health, Yunnan Vocational and Technical College of Agriculture, Kunming 650212, China

## Abstract

Ginsenosides are a class of active components extracted from ginseng plants (such as *Panax ginseng*, *Panax quinquefolium*, and *Panax notoginseng*). Ginsenosides have significant protective effects on the nervous system, cardiovascular system, and immune system, so they have been widely used in the treatment of related diseases. Entry of a variety of endogenous or exogenous harmful substances into the body can lead to an imbalance between the antioxidant defense system and reactive oxygen species, thus producing toxic effects on a variety of tissues and cells. In addition, oxidative stress can alter multiple signaling pathways, including the Keap1/Nrf2/ARE, PI3K/AKT, Wnt/*β*-catenin, and NF-*κ*B pathways. With the deepening of research in this field, various ginsenoside monomers have been reported to exert antioxidant effects through multiple signaling pathways and thus have good application prospects. This article summarized the research advancements regarding the antioxidative effects and related mechanisms of ginsenosides, providing a theoretical basis for experimental research on and clinical treatment with ginsenosides.

## 1. Introduction

Ginseng (*Panax ginseng Meyer*) is one of the most widely used herbal nutrition drugs worldwide. Ginseng has long been used as a dietary supplement and regulator to relieve fatigue in Eastern countries, especially in China, Korea, and Japan [1]. Ginseng has always been regarded as the “king of herbs” in Chinese traditional medicine, as it enhances fitness and tranquilizes the mind. Modern pharmacological studies have suggested that ginseng has various pharmacological effects, including anticancer, antioxidant, anti-inflammatory, and other biological effects [2]. Ginsenosides, which are triterpene saponins, are the major components of ginseng. Thus far, >180 ginsenosides have been isolated from ginseng, and these components have become popular research topics [3]. According to the structures of the glycones, ginsenosides are classified into two major types: dammarane-type ginsenosides and oleanane-type ginsenosides [4]. Based on their chemical structures, dammarane-type ginsenosides are typically further divided into two groups: protopanaxadiol- (PPD-) group ginsenosides and protopanaxatriol- (PPT-) group ginsenosides [5]. The PPD-group ginsenosides include Rb1, Rb2, Rb3, Rc, Rd, Rg3, and Rh2, while the PPT-group ginsenosides include Re, Rg1, Rg2, and Rh1; the oleanane-type ginsenosides mainly includes Ro [6]. These classifications are shown in Figure 1. The biological activities of ginsenosides are influenced by the numbers and locations of sugar molecules, the hydroxyl moieties of the dammarane skeleton, and the stereoisomeric position at C-20 [7]. Research has reported that 20(*R*)-Rg3 shows more potent antioxidant stress activity than 20(*S*)-Rg3 according to the different stereoisomeric positions at C-20 [8]; in addition, 20(*S*)-Rg2 can reduce intracellular UV-B-induced reactive oxygen species (ROS) production and shows more potent antioxidant activity than 20(*R*)-Rg2 [9]. Studies have also found that the secondary metabolite derivatives of ginsenosides after transformation, referred to as rare ginsenosides, have stronger biological activity than the parent compounds [10]. Although the content of these saponins is low, the compounds exhibit unique pharmacological activities. For example, ginsenoside compound K (CK) is an active ginsenoside metabolite of Rb1, Rb2, and Rc that is produced by the intestinal flora after oral administration and can alleviate the cognitive dysfunction associated with vascular dementia in rats [11].

Various ginsenosides can play critical roles in inhibiting oxidative stress, preventing oxidative injury, and protecting cells [12, 13]. However, most of the studies in the literature have focused only on a single signaling pathway, and some relevant studies and reviews do not appear sufficient or comprehensive. Previous reports have tended to review the antioxidant activities of ginsenosides from the perspectives of reducing disease-related symptoms (such as regulating mitochondrial energy metabolism, improving insulin resistance, and reducing complications) [14, 15] and preventing chronic diseases related to oxidative stress (such as diabetes, cancer, and cardiovascular diseases) [16]. However, there have been few reviews about ginsenosides' molecular mechanisms and targets against oxidative stress injury. This review summarizes existing studies on the antioxidant effects, mechanisms, and potential molecular targets of ginsenosides to provide a theoretical basis for the further development of natural antioxidants from ginsenosides.

## 2. Overview of Oxidative Stress

Paniker et al. first proposed the concept of oxidative stress in 1970 when studying the role of glutathione reductase deficiency on the hexose monophosphate shunt pathway under oxidative stress [17]. Oxidative stress is an imbalance between oxidation and antioxidant systems caused by excessive production of ROS or diminished cellular antioxidant activity. Oxidative stress can not only damage macromolecules but also lead to various health disorders, such as atherosclerosis, cancer, neurodegenerative diseases, diabetes mellitus, and obesity [18–22]. Because mitochondria are the primary sources of superoxide free radicals, many previous studies have considered mitochondria the prominent target organelles for oxidative stress [23, 24]. However, at present, oxidative stress is considered a complex biochemical process involving multiple target organelles, such as mitochondria, the Golgi apparatus (GA), the endoplasmic reticulum, and other organelles (Figure 2). When oxidative stress occurs, these organelles can elicit adaptive responses that may protect cells from oxidative injury and restore the oxidation/antioxidant balance [25–27].

Mitochondria are both significant sites of oxygen consumption and the main targets of ROS. The mitochondrial respiratory chain is one of the primary sources of ROS in cells. When oxidative stress injury occurs, mitochondrial dysfunction enhances ROS production, and the damage induced by ROS accumulation can directly or indirectly contribute to mitochondrial dysfunction [28]. The balance of mitochondrial fusion and fission determines mitochondrial morphology and function. Mitochondrial fission is mainly driven by dynamin-related protein 1 (Drp1) and mitochondrial fission protein 1 (Fis1), which primarily mediate mitochondrial division [29]. Mitochondrial fusion is primarily regulated by mitofusins 1 and 2 (Mfn1 and Mfn2) and optic atrophy 1 (Opa1), which have been found to mediate fusion of the outer and inner membranes of mitochondria, respectively [30, 31]. When cells are stimulated by oxidative stress, activation of mitochondrial fission triggers the upregulation of genes associated with BCL2-associated X protein (Bax) and cytochrome C (Cytc), which leads to the fragmentation of mitochondria [32]. Decreased expression of mitochondrial fusion proteins is accompanied by reductions in mitochondrial membrane potential, mitochondrial DNA, and mitochondrial respiratory function, thus causing apoptosis [33].

Endoplasmic reticulum stress (ERS) is caused by the accumulation of misfolded and unfolded proteins in the endoplasmic reticulum (ER) due to disruption of protein processing in the endoplasmic reticulum by pathological factors such as cerebral ischemia-reperfusion injury and oxidative stress [34]. Oxidative stress and ERS interact to induce protein misfolding, leading to ROS production. Overproduction of ROS can disturb the redox homeostasis of the endoplasmic reticulum, disrupt disulfide bond formation, and aggravate protein misfolding and aggregation [35]. In addition, ERS can cause the accumulation of the unfolded protein response (UPR) and disrupt the normal function of the endoplasmic reticulum [36]. When ERS occurs, the balance of endoplasmic reticulum homeostasis is broken, and glucose-regulated protein 78 (GRP78), a transmembrane protein located in the endoplasmic reticulum membrane, elicits the activation of the UPR and causes a range of ERS responses [37]. The activation of ERS can further influence the release and activation of downstream proapoptotic proteins, such as C/EBP homologous protein (CHOP), cysteinyl aspartate specific proteinase-12 (caspase-12), and Bax, and inhibit the expression of the antiapoptotic protein Bcl-2, ultimately leading to apoptosis [38].

The GA considered a “stress sensor” plays crucial roles in Ca^2+^/Mn^2+^ homeostasis, sphingolipid metabolism, and antioxidation. “GA stress” refers to GA-specific stress response [27]. When Ca^2+^/Mn^2+^ homeostasis is imbalanced in GA, the overload of intracellular Ca^2+^ can activate the expression of the caspase family, leading to Golgi fragmentation and apoptosis [39]. It has been reported that the GA can be affected after cerebral ischemia-reperfusion, which may lead to abnormal protein structure and lipid transport, thereby causing physiological dysfunction of neurons [40]. The main pathophysiological processes of GA injuries induced by oxidative stress involve damage to GA tubulin induced by oxidative stress, activation of apoptotic processes of the GA, such as the caspase cascade reaction, and abnormal increases in Ca^2+^ leading to fragmentation of the GA [27]. Golgi phosphoprotein 3 (GOLPH3), the outer membrane protein of the Golgi complex, is involved in many biological processes, including vesicle trafficking, Golgi structure maintenance, and Golgi glycosylation [41]. As a sensor of GA stress, GOLPH3 is rapidly upregulated during oxidative stress and plays a crucial role in GA stress [41]. Li et al. found that GOLPH3 is significantly increased in N2A cells subjected to oxygen-glucose deprivation and reperfusion (OGD/R), which promotes ROS production and leads to apoptosis. In addition, silencing of GOLPH3 with shRNA significantly decreases the apoptosis rate of N2A cells [42]. These findings suggest that oxidative stress in the Golgi can be regulated by the expression of GOLPH3, affecting ROS production.

## 3. Signaling Pathways of Oxidative Stress

During long-term evolution, cells have developed a series of complex mechanisms to cope with oxidative stress involving multiple signaling pathways. These mechanisms produce heme oxygenase 1 (HO-1), glutathione S-transferase (GST), superoxide dismutase (SOD), and other antioxidant substances, which reduce the cellular damage caused by ROS and electrophiles and ultimately maintain the oxidation/antioxidation balance (Figure 3).

### 3.1. Oxidative Stress and the Keap1/Nrf2/ARE Signaling Pathway

When cells are subjected to redox imbalance, they rapidly initiate a variety of antioxidant responses to restore the balance of the redox state. The Kelch-like epoxy chloropropane-related protein-1 (Keap1)/nuclear factor erythroid 2-related factor 2 (Nrf2)/antioxidant response element (ARE) signaling pathway plays a vital role in the amelioration of oxidative stress (Figure 3) [43]. Nrf2 is a crucial redox-sensitive transcription factor in the regulation of multiple cellular antioxidative defenses against both endogenous and exogenous oxidative stress inducers, such as oxidants, exogenous chemical agents, and excessive supply of nutrients/metabolites [44]. As an oxidative stress sensor, Keap1 is inactivated by the oxidation of cysteine residues, which results in the dissociation of Nrf2 from Keap1 [45]. Under normal conditions, Nrf2 is negatively regulated at low levels and undergoes ubiquitin-proteasome degradation through interaction with Keap1. Upon exposure to oxidative stress, the phosphorylation of Nrf2 facilitates the dissociation of Nrf2 from Keap1. Once activated, Nrf2 translocates into the nucleus and binds with the ARE, which promotes the expression of various downstream antioxidant enzymes and exerts antioxidant capacity accordingly [46, 47].

Nrf2 also plays an essential role in maintaining the structural and functional integrity of mitochondria. Under oxidative stress, the activation of Nrf2 can counteract the increase in the production of mitochondrial ROS and maintain the regular function and structure of mitochondria by increasing the activity of antioxidative enzymes, such as glutathione (GSH), SOD, and GST [48, 49]. It has been reported that Nrf2^−/−^ mice are more sensitive to traumatic brain injury- (TBI-) induced oxidative stress than wild-type mice [50]. Choi also found that activation of the Nrf2 signaling pathway can inhibit H_2_O_2_-induced ROS accumulation in human HaCaT keratinocytes, thereby exerting anticytotoxic effects [51]. These experiments indicate that the Nrf2 signaling pathway plays an essential role in inhibiting oxidative stress.

### 3.2. Oxidative Stress and the PI3K/Akt/mTOR Signaling Pathway

The phosphatidylinositol-3-kinase (PI3K)/protein kinase B (Akt) signaling pathway also plays an essential role in the response to oxidative stress, which regulates the cell cycle, proliferation, and apoptosis (Figure 3) [52]. When activated, PI3K catalyzes the production of phosphatidylinositol 3,4,5-triphosphate (PIP3), which binds to phosphorylated Akt in the cytoplasm. The activation of Akt plays an essential role in controlling apoptosis by increasing Bcl-2 expression and decreasing Bax and caspase-3 expression [53]. In addition, the PI3K/Akt signaling pathway might affect the activation of the Nrf2 signaling cascade to promote the expression of antioxidative enzymes [54]. It has been reported that the activation of the PI3K/Akt/Nrf2 signaling pathway can play an antioxidative role, inhibiting apoptosis and alleviating ischemia-reperfusion injury. However, this protective effect is antagonized by LY294002, an inhibitor of the PI3K/Akt signaling pathway [55].

Mammalian target of rapamycin (mTOR), a crucial serine-threonine protein kinase and a major downstream component of the PI3K/Akt signaling pathway, can induce and promote oxidative stress. It has been reported that overactivation of mTOR leads to increased ROS production, while inhibition of mTOR reduces the level of ROS [56]. In addition, mTOR activation can significantly upregulate the expression of the proapoptotic proteins Bax and Bad, which can trigger apoptosis. Furthermore, rapamycin, an inhibitor of mTOR, can protect cells against oxidative stress-induced damage by inhibiting apoptosis [57, 58]. Park et al. proved that an abnormal increase in mTOR could evoke severe oxidative stress, neuroinflammation, and neuronal death in the hippocampus in an animal model of transient ischemia (TI) established in gerbils with high-fat diet- (HFD-) induced obesity [59].

### 3.3. Oxidative Stress and the Wnt/*β*-Catenin Signaling Pathway

It is well known that the Wnt signaling pathway is essential for many fundamental processes of embryonic development and normal tissue homeostasis. The Wnt signaling pathway can be divided into the canonical Wnt pathway (known as the Wnt/*β*-catenin signaling pathway) and the noncanonical Wnt pathway (including the planar cell polarity (PCP) pathway and the Wnt/Ca^2+^ pathway) (Figure 3) [60]. The Wnt/*β*-catenin signaling pathway is mainly composed of the following proteins: *β*-catenin, glycogen synthase kinase-3 (GSK-3), and casein kinase 1 (CK1). Under normal physiological conditions, *β*-catenin is phosphorylated by GSK-3*β* and CK1, and phosphorylated *β*-catenin is targeted for ubiquitination and degradation by the E3-ubiquitin ligase complex. When oxidative stress occurs, GSK-3*β* becomes inactivated by phosphorylation, and *β*-catenin is not degraded; thus, the Wnt/*β*-catenin signaling pathway is activated. Active *β*-catenin translocates from the cytoplasm and accumulates in the nucleus, where it binds to the DNA T-cell transcription factor/lymphatic enhancement transcription factor (TCF/LEF), subsequently promoting the expression of Wnt downstream target genes, such as cMyc, Cyclin D1, and axis inhibition protein 2 (Axin2) [61, 62].

Studies have shown that ethanol-induced oxidative stress can influence mesenchymal stem cell lineage commitment in the bone marrow through downregulation of Wnt/*β*-catenin signaling pathway expression [63]. Experimental animal models of global cerebral ischemia-reperfusion (GCI/R) have demonstrated that activation of the Wnt/*β*-catenin signaling pathway can decrease ROS production. Additionally, the antioxidant effect can be significantly eliminated by using the Wnt signaling pathway inhibitor DDK1 [64].

### 3.4. Oxidative Stress and the NF-*κ*B Signaling Pathway

Nuclear factor-kappa B (NF-*κ*B) is a nuclear transcription factor that plays a critical role in regulating inflammatory responses, cell proliferation, and apoptosis (Figure 3). The NF-*κ*B family of transcription factors consists of five members, including Rel (cRel), p65 (Rel A, NF-*κ*B3), Rel B, p50 (NF-*κ*B1), and p52 (NF-*κ*B2). The NF-*κ*B heterodimer is made up primarily of two subunits, p50 and p65. The activation of NF-*κ*B is involved in the phosphorylation and degradation of inhibitor of NF-*κ*B (I*κ*B) and the release of the NF-*κ*B p65-p50 dimer [65]. In the resting state, NF-*κ*B p50/p65 heterodimers reside inside the cytoplasm in an inactive state and combine with I*κ*B to form a heterotrimer (p50/p65/I*κ*B). When cells are stimulated by NF-*κ*B activators such as tumor necrosis factor-*α* (TNF-*α*) and lipopolysaccharide (LPS), I*κ*B is phosphorylated by I*κ*B kinase (IKK), which results in the degradation of I*κ*B. The dimer of NF-*κ*B is thereby released and translocates into the nucleus, where it can trigger the expression of inflammation-related genes, such as cytokines/chemokines, immune receptors, and cell adhesion molecules [66]. Some studies have shown that doxorubicin (DOX) may increase the inflammatory response in MPC-5 cells by activating the NF-*κ*B signaling pathway, and inhibition of NF-*κ*B activity may alleviate inflammation and oxidative damage [67]. Jin et al. also showed that knockdown of NF-*κ*B with siRNA can exert antioxidant activity and protect against sepsis-induced acute lung injury [68].

### 3.5. Oxidative Stress and Other Signaling Pathways

The occurrence and development of oxidative stress are a very complex process involving multiple signaling pathways. In addition to the pathways mentioned above, other signaling pathways are also involved in oxidative stress, such as the mitogen-activated protein kinase (MAPK) signaling pathway and the transforming growth factor-*β*1 (TGF-*β*1)/Smad signaling pathway. The MAPK signaling pathway is involved in cell survival against oxidative stress and plays an essential role in inflammatory responses. The MAPK signaling pathway is a three-tiered cascade reaction that consists of MAPK kinase kinases (MAPKKKs), MAPK kinases (MAPKKs), and MAPKs [69]. The MAPK family is a family of serine/threonine kinases that includes primarily c-Jun N-terminal kinase (JNK), P38, and extracellular signal-regulated kinases (ERKs). When excessive ROS accumulate, oxidative stress can activate the MAPK signaling pathway, thereby enabling regulated transport of ERK, JNK, and P38 from the cytoplasm to the nucleus; this promotes the transcription and expression of related target genes, causing DNA damage and ultimately leading to apoptosis [70]. In addition, ROS signaling events lead to activation of the TGF-*β*1/Smad signaling pathway [71]. During oxidative stress, TGF-*β*1 increases the generation of ROS and inhibits the activity of antioxidant enzymes, leading to redox imbalance. ROS, in turn, can also activate the expression of TGF-*β*1, and the activated TGF-*β*1 receptor can stimulate the phosphorylation of the Smad protein in the cytoplasm. The activated Smad2/3 protein migrates to the nucleus, resulting in rapid accumulation of the activated complexes, which further exacerbates the imbalance of oxidative stress [72, 73].

## 4. Roles of Ginsenosides and Different Signaling Pathways in the Response to Oxidative Stress

It has been reported that many ginsenoside monomers and their metabolites have antioxidant effects or are potentially involved in regulating many oxidative signaling pathways related to oxidative stress, such as the Keap1/Nrf2/ARE signaling pathway, PI3K/Akt signaling pathway, Wnt/*β*-catenin signaling pathway, and NF-*κ*B signaling pathway.

### 4.1. Ginsenosides Exert Antioxidant Effects through the Keap1/Nrf2/ARE Signaling Pathway

Many studies have reported that various ginsenoside monomers (such as ginsenosides Rg1, Rb1, and Rh3) can exert antioxidant effects by activating the Keap1/Nrf2/ARE signaling pathway. Ning et al. [74] found that ginsenoside Rg1 can inhibit oxidative stress in the liver, as indicated by a decrease in malondialdehyde (MDA) content in the liver and increases in GSH, SOD, and catalase (CAT) content. Ginsenoside Rg1 can also inhibit the liver inflammatory reaction and reduce the expression of TNF-*α*, interleukin-1 beta (IL-1*β*), IL-6, and COX-2, and its potential mechanism of action may be related to the activation of the Nrf2 signaling pathway. Chu et al. [75] found that ginsenoside Rg1 can activate the Nrf2/ARE signaling pathway by inhibiting the expression of miR-144, preventing neuronal injury induced by ischemia-reperfusion *in vivo and in vitro*. Gao et al. [76] demonstrated that ginsenoside Rg1 can protect mice with streptozotocin- (STZ-) induced diabetes against inflammation and oxidative stress by activating the Keap1/Nrf2 pathway. Li et al. [77] confirmed that ginsenoside Rg1 can inhibit hypoxia/reoxygenation- (H/R-) induced H9c2 cell apoptosis and increase the expression of SOD, GSH, and glutathione peroxidase (GSH-Px). The protective effect of ginsenoside Rg1 has been associated with the activation of the Nrf2/HO-1 pathway. Gao et al. [78] found that ginsenoside Rg1 can significantly improve the cell survival rate and reduce excessive ROS and apoptosis by triggering the Nrf2/HO-1 pathway.

Dong et al. [79] demonstrated that ginsenoside Rb1 can reduce the content of MDA and increase the level of GSH and activate the Nrf2 signaling pathway, thereby enabling the expression of downstream antioxidants, such as glutathione cysteine ligase catalytic subunit (GCLC) and glutathione cysteine ligase modulatory subunit (GCLM); these findings suggest that ginsenoside Rb1 can alleviate diabetic retinopathy by regulating the antioxidant function of the rat retina. Jiang et al. [80] confirmed that ginsenoside Rb1 can reduce lung injury in mice after intestinal ischemia-reperfusion by reducing the levels of TNF-*α* and MDA and increasing the expression of Nrf2 and HO-1. Liu et al. [81] found that ginsenoside Rb1 can significantly increase the spinal cord function score, reduce serum MDA content, increase SOD, CAT, and GSH activity, and upregulate Nrf2/HO-1 expression in a spinal cord injury (SCI) rat model. Xu et al. [82] demonstrated that ginsenoside Rh1 promotes proliferation, inhibits apoptosis, and relieves oxidative stress in oxidized low-density lipoprotein- (ox-LDL-) induced vascular endothelial cells (VECs) by activating the Nrf2/HO-1 signaling pathway. Zhang et al. [83] studied the effects of ginsenoside Rg1 on SCI and found that Rg1 could significantly increase the contents of SOD and GSH and inhibit the production of MDA, the potential mechanism of which may be that it exerts antioxidant stress and anti-inflammatory effects by activating Nrf2/HO-1 signaling pathway. Mei et al. [84] found that ginsenoside Rg1 can reduce ROS and MDA contents, restore SOD and GSH-Px activities, and thus inhibit oxidative stress, the mechanism of which is related to the activation of the Nrf2/HO-1 pathway.

Wang et al. [85] found that ginsenoside Rh3 can induce the dissociation of Nrf2 from Keap1, promote the nuclear translocation of Nrf2, and activate the expression of ARE and downstream antioxidant factors in OGD/R-induced endometrial cell injury. Ginsenoside Re, as reported by Liu et al. [86], can reduce ROS production induced by a*β*, maintain mitochondrial function, and inhibit apoptosis. The potential mechanism is related to the activation of the Nrf2 signaling pathway. Zeng et al. [87] found that ginsenoside Rd can improve cardiac function, reduce the infarct area, and reduce the expression of lactate dehydrogenase (LDH) and creatine kinase. Its molecular mechanism of action against myocardial ischemia-reperfusion injury may be partly related to increases in the expression of Nrf2 and HO-1. Yang et al. [88] found that ginsenoside CK can enhance memory function, reduce neuronal apoptosis, increase SOD and GSH levels, reduce MDA content, inhibit a*β* expression, and activate the Keap1/Nrf2/HO-1 signaling pathway in mice with scopolamine-induced memory impairment. These findings suggest that ginsenoside CK has neuroprotective and antioxidant effects *via* activation of the Keap1/Nrf2/HO-1 signaling pathway. Zhao et al. [89] found that the ginsenosides 20(*S*)-Rg3 and 20(*R*)-Rg3 could increase the cell activity and the contents of GSH-Px, SOD, and CAT and decrease activities of LDH, MDA, and ROS on H_2_O_2_-induced H9C2 cells. Meanwhile, further studies showed that 20(*S*)-Rg3 and 20(*R*)-Rg3 could prevent H_2_O_2_-induced oxidative stress injury in H9C2 cells through activating the Keap-1/Nrf2/HO-1 pathway.

### 4.2. Ginsenosides Exert Antioxidant Stress through the PI3K/Akt Signaling Pathway

In addition to the above effects, ginsenosides also exert antioxidant effects by activating the downstream Nrf2 pathway *via* the PI3K/Akt signaling pathway. Chen et al. [90] found that ginsenoside Rb1 can reduce the expression of TNF-*α*, IL-1*β*, IL-6, and MDA in the intestinal tract and increase the expression of SOD, suggesting that ginsenoside Rb1 can attenuate intestinal ischemia-reperfusion-induced inflammation and oxidative stress by activating the PI3K/Akt/Nrf2 signaling pathway. Zhuang et al. [91] studied the antifatigue effect of ginsenoside Rb1 in aged rats with postoperative fatigue syndrome induced by major small intestinal resection (MSIR). Their results showed that ginsenoside Rb1 significantly reduced ROS and MDA release and increased SOD activity in the skeletal muscle of the rats. At the same time, ginsenoside Rb1 increased the mRNA expression of Akt2 and Nrf2, upregulated the phosphorylation of Akt, and promoted the nuclear translocation of Nrf2. Hwang and Jeong [92] found that pretreatment of SH-SY5Y cells with Rb1 significantly reduced 6-hydroxydopamine- (6-OHDA-) induced caspase-3 activation by activating the PI3K/Akt/Nrf2 signaling pathway. In an experiment in which ginsenoside Rg3 was used to inhibit cardiotoxicity induced by adriamycin (ADM), Wang et al. [93] confirmed that Rg3 can attenuate the reduction in the ADM-induced ejection fraction, restore vascular function, promote cell viability, and suppress oxidative damage and apoptosis. Its antioxidant mechanism may be related to the activation of the Akt and Nrf2-ARE pathways. Chen et al. [90] verified that ginsenoside Rb1 can ameliorate intestinal ischemia-reperfusion injury, reduce MDA content, increase SOD levels, and inhibit oxidative stress and the inflammatory response. The molecular mechanism may involve activation of the PI3K/Akt/Nrf2 pathway to improve intestinal ischemia-reperfusion injury. Wortmannin, an inhibitor of PI3K, can inhibit PI3K, which eliminates the protective effect of ginsenoside Rb1. Xiong et al. [94] found that ginsenoside Rk1 significantly improved cell viability, reduced the apoptotic rate, and increased the activity levels of SOD, CAT, and GSH-Px in H_2_O_2_-induced PIG1 cell injury model. These data demonstrated that Rk1protects human melanocytes from H_2_O_2_-induced oxidative injury *via* regulation of the PI3K/AKT/Nrf2/HO-1 pathway.

Nan et al. [95] also confirmed that ginsenoside Rb1 can ameliorate oxidative stress and apoptosis in methylglyoxal- (MGO-) treated SH-SY5Y cells by activating the PI3K/Akt signaling pathway. Li et al. [96] found that 20(*R*)-Rg3 could inhibit the oxidative stress induced by D-gal in the liver and kidney, increase the levels of SOD and CAT, and decrease the levels of MDA and 4-hydroxynonenal (4-HNE). The antioxidative stress effect of 20(*R*)-Rg3 is related to the activation of the PI3K/AKT signaling pathway. Liu et al. [97] found that ginsenoside Rg1 treatment alleviated high glucose-induced oxidative stress by decreasing ROS generation, MDA, and LDH accumulation and increasing the activities of SOD and GSH-Px. The molecular mechanism of Rg1 is considered related to the regulation of the PI3K/AKT/FOXO3 pathway. Xie et al. [98] indicate that ginsenoside Re may ameliorate high glucose-induced retinal angiogenesis and inhibit oxidative stress, and its mechanism of action is associated with the activation of the PI3K/AKT signaling pathway.

It has been confirmed that ginsenosides can also act on the classical PI3K/Akt/mTOR signaling pathway and exert antioxidant effects by downregulating the Akt/mTOR pathway. Chen et al. [99] found that ginsenoside Rg1 improved cognitive impairment induced by D-gal in mice by attenuating the senescence of neural stem cells. Rg1 also decreased the level of oxidative stress, increasing the activity of SOD and GSH-Px, *in vivo* and *in vitro.* Rg1 further reduced the phosphorylation levels of Akt and mTOR. These findings suggested that the ginsenoside Rg1-mediated attenuation of cognitive impairment in mice and senescence in neural stem cells (NSCs) induced by D-gal might have been related to a reduction in oxidative stress and downregulation of the Akt/mTOR signaling pathway.

### 4.3. Ginsenosides Exert Antioxidant Stress through the Wnt/*β*-Catenin Signaling Pathway

Wnt signaling is closely related to oxidative stress. Oxidative stress induced by various factors inhibits the Wnt/*β*-Catenin signaling pathway. Ginsenoside intervention can activate the Wnt/*β*-Catenin signaling pathway and reduce the damage caused by oxidative stress. Li et al. [100] explored the protective effect of ginsenoside Rg1 on hematopoietic stem cells in a mouse model of D-gal-induced aging. The results showed that Rg1 exerted antioxidant stress by reducing the levels of ROS and MDA and increasing the total antioxidant capacity (T-AOC) and the expression of SOD and GSH-px. The mechanism might have been related to the activation of the Wnt/*β*-catenin signaling pathway. Zu et al. [101] found that ginsenoside Rg1 can inhibit intestinal ischemia-reperfusion injury through a molecular mechanism also related to activation of the Wnt/*β*-catenin signaling pathway, inhibition of ROS, and suppression of apoptosis. Shao et al. [102] found that ginsenoside Rb1 can significantly reduce renal dysfunction, oxidative stress, and pathological changes in rats with streptozotocin-induced diabetic nephropathy through a mechanism related to the regulation of miR-350 expression and further activation of the Wnt/*β*-catenin signaling pathway. In conclusion, ginsenosides can play antioxidant roles by activating the Wnt/*β*-Catenin signaling pathway via upregulation of SOD and GSH-Px expression, upregulation of T-AOC, and downregulation of ROS and MDA levels.

### 4.4. Ginsenosides Exert Antioxidant Effects through the NF-*κ*B Signaling Pathway

The transcription factor NF-*κ*B is widely expressed and regulates various cellular processes, including inflammation, immune response processes, cell proliferation, and apoptosis [66]. During oxidative stress, activation of the NF-*κ*B signaling pathway can induce tissue damage. In recent years, it has been reported that ginsenosides can protect tissue from oxidative stress by inhibiting the NF-*κ*B signaling pathway [103]. Ye et al. [104] studied the effect of ginsenoside Rg1 on rats with lung injury induced by hindlimb ischemia-reperfusion. The results confirmed that Rg1 alleviated lung injury by inhibiting the NF-*κ*B/cyclooxygenase-2 (COX-2) signaling pathway. Song et al. [105] found that ginsenoside CK had a protective effect against diabetes-induced renal injury. Ginsenoside CK inhibited diabetes-induced oxidative stress by downregulating the expression of nicotinamide adenine dinucleotide phosphate (NADPH) oxidase and inhibiting the NF-*κ*B/p38 signaling pathway. Hou and Kim [106] used H_2_O_2_ to establish a senescence model in human dermal fibroblasts and found that ginsenoside Rb1 enhanced dermal fibroblast differentiation in aging skin and promoted skin wound healing by inhibiting the p38MAPK/MSK2/NF-*κ*B pathway. Chen et al. [107] studied the protective effect of ginsenoside Rg3 on TNF-*α*-treated human nucleus pulposus cells (NPCs) and found that Rg3 reduced ROS and MDA levels, increased GSH-px and SOD expression, and inhibited apoptosis. The mechanism may have been related to the blockade of the NF-*κ*B signaling pathway. Li et al. [108] found that 20(*R*)-ginsenoside Rg3 ameliorated diabetic nephropathy in mice by improving antioxidant activity and reducing renal inflammation. 20(*R*)-Rg3 reduced MDA levels and increased SOD and CAT production through a mechanism related to inhibition of the MAPK/NF-*κ*B signaling pathway. Hou et al. [109] studied the effects of ginsenoside Rh2 on adriamycin-induced cell senescence in breast cancer and normal epithelial cells and confirmed that ginsenoside Rh2 reduced ROS production, increased SOD expression, reduced oxidative stress, and inhibited the NF-*κ*B signaling pathway in senescent cells. Chen et al. [107] found that ginsenoside Rg3 can reduce TNF-*α*-induced damage to human NPCs by blocking the NF-*κ*B signaling pathway. Ginsenoside Rg3 can also reduce the production of ROS and MDA, increase the activity of SOD and GSH-Px, and reduce the cell damage induced by oxidative stress. Ren et al. [110] demonstrated that ginsenoside Rg3 prevents angiotensin II- (Ang II-) induced myocardial hypertrophy *via* inactivating NLRP3 inflammasome and oxidative stress by modulating the NF-*κ*B pathway. Zhu et al. [111] investigated the effect of Rg5 on kidney injury of C57BL/6 diabetic mice induced by high-fat diet and streptozotocin, and the results showed that Rg5 decreased the production of ROS and MDA, increased the activities of SOD and GSH-Px, and inhibited the activation of NF-*κ*B signaling pathway.

### 4.5. Ginsenosides Exert Antioxidant Effects through Other Signaling Pathways

In addition to the above signaling pathways, ginsenosides can also exert antioxidant effects by influencing different signaling pathways. Zhou et al. [112] reported that ginsenosides have a strong protective effect on the cholinergic nervous system in rats with acute renal failure (ARF) induced by myoglobin release. Their findings confirmed that ginsenosides can reduce oxidative stress in the kidneys that is related to the activation of the MAPK signaling pathway. Chen et al. [113] found that in Parkinson's disease mice, ginsenoside Rg1 prevented loss of substantia nigra neurons, inhibited decreases in GSH and T-SOD in the substantia nigra, and inhibited phosphorylation of JNK and c-Jun. Zhou et al. [114] found that ginsenoside Rb1 has a protective effect against endothelial cell injury induced by TNF-*α*. Specifically, they confirmed that Rb1 can inhibit the production of ROS and MDA induced by TNF-*α*; increase the activity of SOD, CAT, and GSH-Px; and protect endothelial cells from oxidative stress and inflammation induced by TNF-*α* by inhibiting NF-*κ*B, JNK, and p38. Cong and Cheng [115] evaluated the neuroprotective effect of ginsenoside Rd in a rat model of SCI and found that ginsenoside Rd decreased MDA expression and increased GSH and SOD expression. Ginsenoside Rd also improved motor function, increased the survival rate of spinal cord neurons, and reduced tissue injury by inhibiting the MAPK signaling pathway. Zhang et al. [116] found that ginsenoside Rb1 can reduce ROS production, inhibit the expression of NOX subtypes NOX1 and NOX4, and downregulate the expression of NADPH oxidase induced by diabetes mellitus (DM), and the mechanism is related to the inhibition of the TGF*β*1/Smad2/3 pathway.

Combinations of various ginsenosides can enhance the antioxidant effects of these compounds. The combination of PPT and Rb1 or Rg1 has synergistic antioxidant activity, and its mechanism is related to the activation of the Nrf2-ARE signaling pathway [117]. In addition, combining ginsenosides with other active ingredients can lead to synergistic effects, enhancing the antioxidant functions of the ginsenosides. For example, combining pumpkin polysaccharide with ginsenoside Rg1 can significantly improve the activity of this ginsenoside against H_2_O_2_-induced oxidative stress in cells, reduce the levels of MDA in cells, and significantly reduce lipid peroxidation damage in cells. By increasing the activity of SOD, GST-px, and CAT in cells, pumpkin polysaccharide, and ginsenoside Rg1 show good antioxidant activity and ameliorate oxidative stress damage in cells. Du et al. [118] studied the effects of the combined application of ginsenoside Rg1 and astragaloside IV on oxidative stress in a rat model of diabetic nephropathy. The results confirmed that both ginsenoside Rg1 and astragaloside IV had antioxidant effects. Their combined application enhanced T-AOC, possibly via inhibition of TGF-beta 1/Smad cascade signaling.

## 5. Summary and Future Perspectives

Research on the effects of ginsenosides' antioxidant stress has made great progress in recent years. Based on the published literature, the main active components of ginseng play an important role in protecting multiple organelles from oxidative stress, which may be related to the regulation of various signaling pathways, such as the Keap1/Nrf2/ARE, PI3K/Akt, Wnt/*β*-catenin, NF-*κ*B, and other signaling pathways (Table 1). Although the antioxidant effects of ginsenosides and their monomers have been widely reported, many potential mechanisms of antioxidant stress and the pharmacological effects of ginsenosides have not been fully elucidated. The majority of the existing research on the pharmacological effects of ginsenosides was isolated and needs more in-depth and extensive investigations. Second, most of the studies on the pharmacological effects of ginsenosides focus on animal and/or cellular levels, and associated evaluation of the clinical applications has rarely been performed. Therefore, it is necessary to carry out such studies to verify the clinical efficacy of ginsenosides on antioxidant stress. In addition, further work is needed to elucidate the underlying mechanism of action, pharmacokinetics, and pharmacodynamics of the main active ingredients in ginsenosides, to provide more theoretical and experimental bases for clinic interventions.

## Figures and Tables

**Figure 1:** Structures of main ginsenosides. The figure shows the molecular structure of 20(*R*)-ginsenosides and 20(*S*)-ginsenosides. The main difference between them that is R1, R2, and R3 form a glycoside position (glc: *β*-d-glucopyranoside; ara (pyr): arabinopyranoside; ara (fur): furanoside; xyl: xylose group; rha: rhamnose).

**Figure 2:** Schematic diagram of multiple damaged organelles induced by oxidative stress. The figure shows that oxidative stress can cause apoptosis and the changes of mitochondria, GA, and ER after oxidative stress. Oxidative stress can lead to abnormal mitochondrial fusion division, dysfunction of the endoplasmic reticulum, imbalance of Golgi Ca^2+^ homeostasis, and Golgi fragmentation.

**Figure 3:** The schematic overview of major signaling pathways induced by oxidative stress. The overproduction of ROS leads to the imbalance of oxidation/antioxidants, which causes various signaling pathways to regulate the process of oxidative stress. Activation of Keap1/Nrf2/ARE and PI3K/Akt signaling pathways can induce the expression of antioxidants and play an antioxidative stress role. In addition, mTOR, Wnt/*β*-catenin, and NF-*κ*B signaling pathways are also involved in the process of oxidative stress, and inhibition of these signaling pathways may play a protective role against oxidative stress.

**Table 1:** Antioxidant stress effects of ginsenosides *in vivo* and *in vitro*.

Disease model	Cell line	Ginsenoside type	Signal pathway	Antioxidant biomarker	Ref
CCl_4_-induced acute liver injury	Without	Rg1	Nrf2	MDA↓, GSH↑, SOD↑, CAT↑	[74]
tMCAO	PC12	Rg1	Nrf2-ARE	ROS↓, HO-1↑, GCLC↑, GCLM↑, NQO-1↑	[75]
Without	Hypoxia/reoxygenation–induced H9c2 cells	Rg1	Nrf2/HO-1	SOD↑, GSH↑, GSH-Px↑	[77]
Diabetic retinopathy in streptozotocin-induced diabetic rats	Without	Rb1	Nrf2	MDA↓, GSH↑, GCLC↑, GCLM↑	[79]
Intestinal ischemia/reperfusion	Without	Rb1	Nrf2/HO-1	MDA↓, TNF-*α*↓, SOD↑, HO-1↑	[80]
Spinal cord injury	Without	Rb1	eNOS/Nrf2/HO-1	MDA↓, SOD↑, CAT↑, GSH↑	[81]
Without	Ox-LDL-treated VECs	Rh1	Nrf2/HO-1	ROS↓, MDA↓, SOD↑	[82]
Rat SCI model	Without	Rg1	Nrf2/HO-1	MDA↓, SOD↑, GSH↑	[83]
SAE mouse model	Mouse neuron cells and microglia BV2 cells	Rg1	Nrf2/HO-1	MDA↓, SOD↑, GSH-Px↑	[84]
Myocardial ischemia-reperfusion	Without	Rd	Nrf2/HO-1	CK↓, LDH↓, HO-1↑	[87]
Without	H_2_O_2_-induced H9C2 cells	20(*S*)-Rg3 and 20(*R*)-Rg3	Keap1/Nrf2/HO-1	ROS↓, MDA↓, SOD↑, GSH-Px↑, CAT↑	[89]
Intestinal ischemia/reperfusion	Without	Rb1	PI3K/Akt/Nrf2	MDA↓, TNF-*α*↓, IL-1*β*↓, IL-6↓, SOD↑	[90]
Postoperative fatigue syndrome	Without	Rb1	PI3K/Akt/Nrf2	ROS↓, MDA↓, SOD↑	[91]
Without	6-OHDA-induced SH-SY5Y	Rb1	PI3K/AKT/Nrf2	HO-1↑, caspase↓	[92]
Adriamycin-induced cardiotoxicity	Endothelial	Rg3	Nrf2-ARE	ROS↓, MDA↓, SOD↑, eNOS↑	[93]
Without	H_2_O_2_- induced melanocytes	Rk1	PI3K/AKT/Nrf2/HO-1	SOD↑, GSH-Px↑, CAT↑	[94]
D-gal-induced in mice	Without	20(*R*)-Rg3	PI3K/AKT	MDA↓, 4-HNE↓, SOD↑, CAT↑	[96]
DN rat model	HG-induced HBZY-1 cells	Rg1	PI3K/AKT/FOXO3	ROS↓, MDA↓, SOD↑, GSH-Px↑	[97]
Without	Hyperglycaemia-induced endothelial cell	Re	PI3K/AKT	ROS↓, MDA↓, GSH-Px↑, CAT↑	[98]
D-gal-induced in mice	NSCs	Rg1	Akt/mTOR	SOD↑, GSH-Px↑	[99]
Without	Hematopoietic stem cell	Rg1	Wnt/*β*-catenin	ROS↓, MDA↓, SOD↑, GSH-Px↑, T-AOC↑	[100]
Intestinal ischemia/reperfusion	Without	Rg1	Wnt/*β*-catenin	ROS↓, MDA↓, SOD↑, GSH↑	[101]
Hind-limb IR	Without	Rg1	NF-*κ*B	MPO↑, SOD↑, CAT↑, NF-*κ*B↓, COX-2↓	[104]
Diabetic nephropathy	Without	CK	NF-*κ*B	ROS↓, IL-1*β*↓	[105]
Without	Human dermal fibroblast	Rb1	NF-*κ*B	TGF-*β*↓, VEGF↑, p38↓	[106]
Without	TNF-*α* induced human nucleus pulposus cells	Rg3	NF-*κ*B	ROS↓, MDA↓, SOD↑, GSH-Px↑	[107]
Myocardial hypertrophy model in rats	Ang II-induced AC16 and HCM cells	Rg3	NF-*κ*B	MDA↓, SOD↑	[110]
DN mice	Without	Rg5	MAPK	ROS↓, MDA↓, SOD↑, GSH-Px↑	[111]
Glycerol-induced acute renal failure in rats	Without	GS	MAPK	MDA↓, SOD↑	[112]
MPTP-induced Parkinson's disease mice	Without	Rg1	JNK	T-SOD↑, GSH↑	[113]
Without	TNF-*α*-induced endothelial cell injury	Rb1	NF-*κ*B, JNK, p38	ROS↓, MDA↓, SOD↑, CAT↑, GSH-Px↑	[114]
Spinal cord injury rats	Without	Rd	MAPK	MDA↓, SOD↑, GSH↑, IL-1*β*↓, IL-1↓	[115]
Streptozotocin-induced mices	Without	Rb1	TGF*β*1/Smad2/3	ROS↓, NOX1↓, NOX4↓	[116]
Diabetic nephropathy rats	Without	Rg1 and astragaloside IV	TGF-*β*1/Smads	MDA↓, CAT↑, GSH-Px↑, T-AOC↑	[118]

## Abbreviations

PPD: Protopanaxadiol
PPT: Protopanaxatriol
ROS: Reactive oxygen species
CK: Ginsenoside compound K
GA: Golgi apparatus
Drp1: Dynamin-related protein 1
Fis1: Mitochondrial fission protein 1
Mfn1/Mfn2: Mitofusins 1 and 2
Opa1: Optic atrophy 1
Bax: BCL2-associated X protein
Cytc: Cytochrome C
ERS: Endoplasmic reticulum stress
ER: Endoplasmic reticulum
UPR: Unfolded protein response
GRP78: Glucose-regulated protein 78
CHOP: C/EBP homologous protein
GOLPH3: Golgi phosphoprotein-3
OGD/R: Oxygen-glucose deprivation and reperfusion
Caspase: Cysteinyl aspartate specific proteinase
HO-1: Heme oxygenase 1
GST: Glutathione S-transferase
SOD: Superoxide dismutase
Keap1: Kelch-like epoxy chloropropane-related protein-1
Nrf2: Nuclear factor erythroid 2-related factor 2
ARE: Antioxidant response element
GSH: Glutathione
TBI: Traumatic brain injury
PI3K: Phosphatidylinositol-3-kinase
Akt: Protein kinase B
PIP3: Phosphatidylinositol 3,4,5-triphosphate
mTOR: Mammalian target of rapamycin
TI: Transient ischemia
HFD: High-fat diet
PCP: Planar cell polarity
GSK-3: Glycogen synthase kinase-3
CK1: Casein kinase 1
TCF/LEF: DNA T-cell transcription factor/lymphatic enhancement transcription factor
Axin2: Axis inhibition protein 2
GCI/R: Global cerebral ischemia-reperfusion
NF-*κ*B: Nuclear factor-kappa B
I*κ*B: Inhibitor of NF-*κ*B
TNF-*α*: Tumor necrosis factor-*α*
LPS: Lipopolysaccharide
IKK: I*κ*B kinase
DOX: Doxorubicin
MAPK: Mitogen-activated protein kinase
TGF-*β*1: Transforming growth factor-*β*1
MAPKKs: MAPK kinases
MAPKKKs: MAPK kinase kinases
JNK: c-Jun N-terminal kinase
ERKs: Extracellular signal-regulated kinases
MDA: Malondialdehyde
CAT: Catalase
IL-1*β*: Interleukin-1 beta
STZ: Streptozotocin
H/R: Hypoxia/reoxygenation
GSH-Px: GSH and glutathione peroxidase
GCLC: Glutathione cysteine ligase catalytic subunit
GCLM: Glutathione cysteine ligase modulatory subunit
SCI: Spinal cord injury
ox-LDL: Oxidized low-density lipoprotein
VECs: Vascular endothelial cells
LDH: Lactate dehydrogenase
MSIR: Major small intestinal resection
6-OHDA: 6-Hydroxydopamine
ADM: Adriamycin
D-gal: D-galactose
4-HNE: 4-Hydroxynonenal
DN: Diabetic nephropathy
HG: High glucose
NSCs: Neural stem cells
T-AOC: Total antioxidant capacity
COX-2: Cyclooxygenase-2
NADPH: Nicotinamide adenine dinucleotide phosphate
NPCs: Nucleus pulposus cells
Ang II: Angiotensin II
NLRP3: NACHT, LRR, and PYD domains-containing protein 3
ARF: Acute renal failure
DM: Diabetes mellitus
NQO1: NAD(P)H quinone dehydrogenase 1
iNOS: Inducible nitric oxide synthase
TNF-*β*: Tumor necrosis factor-*β*
SAE: Sepsis-associated encephalopathy.

## References

[1] Shi Z. Y., Zeng J. Z., Wong A. S. T. (2019). Chemical structures and pharmacological profiles of ginseng saponins. *Molecules*.

[2] Metwaly A. M., Lianlian Z., Luqi H., Deqiang D. (2019). Black ginseng and its saponins: preparation, phytochemistry and pharmacological effects. *Molecules*.

[3] Yu S. E., Mwesige B., Yi Y. S., Yoo B. C. (2019). Ginsenosides: the need to move forward from bench to clinical trials. *Journal of Ginseng Research*.

[4] He Y., Hu Z., Li A. (2019). Recent advances in biotransformation of saponins. *Molecules*.

[5] Kim Y. J., Zhang D., Yang D. C. (2015). Biosynthesis and biotechnological production of ginsenosides. *Biotechnology Advances*.

[6] Choi W. Y., Lim H. W., Lim C. J. (2013). Anti-inflammatory, antioxidative and matrix metalloproteinase inhibitory properties of 20(R)-ginsenoside Rh2 in cultured macrophages and keratinocytes. *The Journal of Pharmacy and Pharmacology*.

[7] Cheong J. H., Kim H., Hong M. J. (2015). Stereoisomer-specific anticancer activities of ginsenoside Rg3 and Rh2 in HepG2 cells: disparity in cytotoxicity and autophagy-inducing effects due to 20(S)-epimers. *Biological & Pharmaceutical Bulletin*.

[8] Li G., Zhang X.-X., Lin L. (2014). Preparation of ginsenoside Rg3 and protection against H2O2-induced oxidative stress in human neuroblastoma SK-N-SH cells. *Journal of Chemistry*.

[9] Kang H. J., Huang Y. H., Lim H. W. (2016). Stereospecificity of ginsenoside Rg2 epimers in the protective response against UV-B radiation-induced oxidative stress in human epidermal keratinocytes. *Journal of Photochemistry and Photobiology. B*.

[10] Zheng M. M., Xu F. X., Li Y. J. (2017). Study on transformation of ginsenosides in different methods. *BioMed Research International*.

[11] Zong W., Zeng X., Chen S. (2019). Ginsenoside compound K attenuates cognitive deficits in vascular dementia rats by reducing the A*β* deposition. *Journal of Pharmacological Sciences*.

[12] Ong W. Y., Farooqui T., Koh H. L., Farooqui A. A., Ling E. A. (2015). Protective effects of ginseng on neurological disorders. *Frontiers in Aging Neuroscience*.

[13] Kang K. S., Ham J., Kim Y. J., Park J. H., Cho E. J., Yamabe N. (2013). Heat-processed Panax ginseng and diabetic renal damage: active components and action mechanism. *Journal of Ginseng Research*.

[14] Zhou P., Xie W., Sun Y. (2019). Ginsenoside Rb1 and mitochondria: a short review of the literature. *Molecular and Cellular Probes*.

[15] Zhou P., Xie W., He S. (2019). Ginsenoside Rb1 as an anti-diabetic agent and its underlying mechanism analysis. *Cell*.

[16] Lee Y. M., Yoon H., Park H. M., Song B. C., Yeum K. J. (2017). Implications of red _Panax ginseng_ in oxidative stress associated chronic diseases. *Journal of Ginseng Research*.

[17] Paniker N. V., Srivastava S. K., Beutler E. (1970). Glutathione metabolism of the red cells effect of glutathione reductase deficiency on the stimulation of hexose monophosphate shunt under oxidative stress. *Biochimica et Biophysica Acta*.

[18] Ray P. D., Huang B. W., Tsuji Y. (2012). Reactive oxygen species (ROS) homeostasis and redox regulation in cellular signaling. *Cellular Signalling*.

[19] Chen Z., Zhong C. (2014). Oxidative stress in Alzheimer's disease. *Neuroscience Bulletin*.

[20] Bisht S., Faiq M., Tolahunase M., Dada R. (2017). Oxidative stress and male infertility. *Nature Reviews. Urology*.

[21] Senoner T., Dichtl W. (2019). Oxidative stress in cardiovascular diseases: still a therapeutic target?. *Nutrients*.

[22] Costa C., Tsatsakis A., Mamoulakis C. (2017). Current evidence on the effect of dietary polyphenols intake on chronic diseases. *Food and Chemical Toxicology*.

[23] Gil J., Almeida S., Oliveira C. R., Rego A. C. (2003). Cytosolic and mitochondrial ROS in staurosporine-induced retinal cell apoptosis. *Free Radical Biology & Medicine*.

[24] Ungurianu A., Seremet O., Gradinaru D., Ionescu-Tirgoviste C., Margina D., Dănciulescu Miulescu R. (2019). Spectrophotometric versus spectrofluorometric assessment in the study of the relationships between lipid peroxidation and metabolic dysregulation. *Chemical Biology & Drug Design*.

[25] Ott M., Gogvadze V., Orrenius S., Zhivotovsky B. (2007). Mitochondria, oxidative stress and cell death. *Apoptosis*.

[26] Bhandary B., Marahatta A., Kim H. R., Chae H. J. (2013). An involvement of oxidative stress in endoplasmic reticulum stress and its associated diseases. *International Journal of Molecular Sciences*.

[27] Jiang Z., Hu Z., Zeng L. (2011). The role of the Golgi apparatus in oxidative stress: is this organelle less significant than mitochondria?. *Free Radical Biology & Medicine*.

[28] Park J., Lee J., Choi C. (2011). Mitochondrial network determines intracellular ROS dynamics and sensitivity to oxidative stress through switching inter-mitochondrial messengers. *PLoS One*.

[29] Elgass K., Pakay J., Ryan M. T., Palmer C. S. (2013). Recent advances into the understanding of mitochondrial fission. *Biochimica et Biophysica Acta*.

[30] Cho D. H., Nakamura T., Lipton S. A. (2010). Mitochondrial dynamics in cell death and neurodegeneration. *Cellular and Molecular Life Sciences*.

[31] Saita S., Ishihara T., Maeda M. (2016). Distinct types of protease systems are involved in homeostasis regulation of mitochondrial morphology via balanced fusion and fission. *Genes to Cells*.

[32] Youle R. J., Karbowski M. (2005). Mitochondrial fission in apoptosis. *Nature Reviews. Molecular Cell Biology*.

[33] Bossy-Wetzel E., Barsoum M. J., Godzik A., Schwarzenbacher R., Lipton S. A. (2003). Mitochondrial fission in apoptosis, neurodegeneration and aging. *Current Opinion in Cell Biology*.

[34] Maamoun H., Benameur T., Pintus G., Munusamy S., Agouni A. (2019). Crosstalk between oxidative stress and endoplasmic reticulum (ER) stress in endothelial dysfunction and aberrant angiogenesis associated with diabetes: a focus on the protective roles of heme oxygenase (HO)-1. *Frontiers in Physiology*.

[35] Wang J., Yang X., Zhang J. (2016). Bridges between mitochondrial oxidative stress, ER stress and mTOR signaling in pancreatic *β* cells. *Cellular Signalling*.

[36] Rutkowski D. T., Kaufman R. J. (2004). A trip to the ER: coping with stress. *Trends in Cell Biology*.

[37] Ron D., Walter P. (2007). Signal integration in the endoplasmic reticulum unfolded protein response. *Nature Reviews. Molecular Cell Biology*.

[38] Li Y., Guo Y., Tang J., Jiang J., Chen Z. (2014). New insights into the roles of CHOP-induced apoptosis in ER stress. *Acta Biochim Biophys Sin (Shanghai).*.

[39] Ji G., Ji H., Mo X., Li T., Yu Y., Hu Z. (2013). The role of GRASPs in morphological alterations of Golgi apparatus: mechanisms and effects. *Reviews in the Neurosciences*.

[40] Vanoevelen J., Raeymaekers L., Dode L. (2005). Cytosolic Ca^2+^ signals depending on the functional state of the Golgi in HeLa cells. *Cell Calcium*.

[41] Li T., You H., Zhang J. (2014). Study of GOLPH3: a potential stress-inducible protein from Golgi apparatus. *Molecular Neurobiology*.

[42] Li T., You H., Mo X. (2016). GOLPH3 mediated Golgi stress response in modulating N2A cell death upon oxygen-glucose deprivation and reoxygenation injury. *Molecular Neurobiology*.

[43] Loboda A., Damulewicz M., Pyza E., Jozkowicz A., Dulak J. (2016). Role of Nrf2/HO-1 system in development, oxidative stress response and diseases: an evolutionarily conserved mechanism. *Cellular and Molecular Life Sciences*.

[44] Dai X., Yan X., Wintergerst K. A., Cai L., Keller B. B., Tan Y. (2020). Nrf2: redox and metabolic regulator of stem cell state and function. *Trends in Molecular Medicine*.

[45] Yamamoto M., Kensler T. W., Motohashi H. (2018). The KEAP1-NRF2 system: a thiol-based sensor-effector apparatus for maintaining redox homeostasis. *Physiological Reviews*.

[46] Bellezza I., Giambanco I., Minelli A., Donato R. (2018). Nrf2-Keap1 signaling in oxidative and reductive stress. *Biochim Biophys Acta Mol Cell Res.*.

[47] Leung C. H., Zhang J. T., Yang G. J., Liu H., Han Q. B., Ma D. L. (2019). Emerging screening approaches in the development of Nrf2-Keap1 protein-protein interaction inhibitors. *International Journal of Molecular Sciences*.

[48] Dinkova-Kostova A. T., Abramov A. Y. (2015). The emerging role of Nrf2 in mitochondrial function. *Free Radical Biology & Medicine*.

[49] Sabouny R., Fraunberger E., Geoffrion M. (2017). The Keap1-Nrf2 stress response pathway promotes mitochondrial hyperfusion through degradation of the mitochondrial fission protein Drp1. *Antioxidants & Redox Signaling*.

[50] Zhang M., Huang L. L., Teng C. H. (2018). Isoliquiritigenin provides protection and attenuates oxidative stress-induced injuries via the Nrf2-ARE signaling pathway after traumatic brain injury. *Neurochemical Research*.

[51] Choi Y. H. (2019). Activation of the Nrf2/HO-1 signaling pathway contributes to the protective effects of coptisine against oxidative stress-induced DNA damage and apoptosis in HaCaT keratinocytes. *General Physiology and Biophysics*.

[52] Xie Y., Shi X., Sheng K. (2019). PI3K/Akt signaling transduction pathway, erythropoiesis and glycolysis in hypoxia (review). *Molecular Medicine Reports*.

[53] Huang X., Liu G., Guo J., Su Z. (2018). The PI3K/AKT pathway in obesity and type 2 diabetes. *International Journal of Biological Sciences*.

[54] Wang L., Chen Y., Sternberg P., Cai J. (2008). Essential roles of the PI3 kinase/Akt pathway in regulating Nrf2-dependent antioxidant functions in the RPE. *Investigative Ophthalmology & Visual Science*.

[55] Wen Z., Hou W., Wu W. (2018). 6-O-Galloylpaeoniflorin Attenuates Cerebral Ischemia Reperfusion-Induced Neuroinflammation and Oxidative Stress via PI3K/Akt/Nrf2 Activation. *Oxidative Medicine and Cellular Longevity*.

[56] Kim J. H., Chu S. C., Gramlich J. L. (2005). Activation of the PI3K/mTOR pathway by BCR-ABL contributes to increased production of reactive oxygen species. *Blood*.

[57] Lu Q., Zhou Y., Hao M. (2018). The mTOR promotes oxidative stress-induced apoptosis of mesangial cells in diabetic nephropathy. *Molecular and Cellular Endocrinology*.

[58] Kocak Z., Temiz-Resitoglu M., Guden D. S. (2019). Modulation of oxidative–nitrosative stress and inflammatory response by rapamycin in target and distant organs in rats exposed to hindlimb ischemia–reperfusion: the role of mammalian target of rapamycin. *Canadian Journal of Physiology and Pharmacology*.

[59] Park J. H., Ahn J. H., Song M. (2019). A 2-min transient ischemia confers cerebral ischemic tolerance in non-obese gerbils, but results in neuronal death in obese gerbils by increasing abnormal mTOR activation-mediated oxidative stress and neuroinflammation. *Cell*.

[60] Katoh M., Katoh M. (2007). WNT signaling pathway and stem cell signaling network. *Clinical Cancer Research*.

[61] Bem J., Brozko N., Chakraborty C. (2019). Wnt/*β*-catenin signaling in brain development and mental disorders: keeping TCF7L2 in mind. *FEBS Letters*.

[62] Kahn M. (2014). Can we safely target the WNT pathway?. *Nature Reviews. Drug Discovery*.

[63] Chen J. R., Lazarenko O. P., Shankar K., Blackburn M. L., Badger T. M., Ronis M. J. (2010). A role for ethanol-induced oxidative stress in controlling lineage commitment of mesenchymal stromal cells through inhibition of Wnt/*β*-catenin signaling. *Journal of Bone and Mineral Research*.

[64] Tang Y., Shen J., Zhang F., Yang F. Y., Liu M. (2019). Human serum albumin attenuates global cerebral ischemia/reperfusion-induced brain injury in a Wnt/*β*-catenin/ROS signaling-dependent manner in rats. *Biomedicine & Pharmacotherapy*.

[65] Dresselhaus E. C., Meffert M. K. (2019). Cellular specificity of NF-*κ*B function in the nervous system. *Frontiers in Immunology*.

[66] Queisser N., Schupp N. (2012). Aldosterone, oxidative stress, and NF-*κ*B activation in hypertension-related cardiovascular and renal diseases. *Free Radical Biology & Medicine*.

[67] Zhu M. M., Wang L., Yang D. (2019). Wedelolactone alleviates doxorubicin-induced inflammation and oxidative stress damage of podocytes by I*κ*K/I*κ*B/NF-*κ*B pathway. *Biomedicine & Pharmacotherapy*.

[68] Jin L. Y., Li C. F., Zhu G. F., Wu C. T., Wang J., Yan S. F. (2014). Effect of siRNA against NF-*κ*B on sepsis-induced acute lung injury in a mouse model. *Molecular Medicine Reports*.

[69] Jalmi S. K., Sinha A. K. (2015). ROS mediated MAPK signaling in abiotic and biotic stress- striking similarities and differences. *Frontiers in Plant Science*.

[70] Soga M., Matsuzawa A., Ichijo H. (2012). Oxidative stress-induced diseases via the ASK1 signaling pathway. *International journal of cell biology*.

[71] Lv W., Booz G. W., Fan F., Wang Y., Roman R. J. (2018). Oxidative stress and renal fibrosis: recent insights for the development of novel therapeutic strategies. *Frontiers in Physiology*.

[72] Liu R. M., Desai L. P. (2015). Reciprocal regulation of TGF-*β* and reactive oxygen species: a perverse cycle for fibrosis. *Redox Biology*.

[73] Li C., Sun X., Li A., Mo M., Zhao Z. (2020). S-Allylmercaptocysteine attenuates bleomycin-induced pulmonary fibrosis in mice via suppressing TGF-*β*1/Smad and oxidative stress pathways. *International Immunopharmacology*.

[74] Ning C., Gao X., Wang C. (2018). Hepatoprotective effect of ginsenoside Rg1 from Panax ginseng on carbon tetrachloride-induced acute liver injury by activating Nrf2 signaling pathway in mice. *Environmental Toxicology*.

[75] Chu S. F., Zhang Z., Zhou X. (2019). Ginsenoside Rg1 protects against ischemic/reperfusion-induced neuronal injury through miR-144/Nrf2/ARE pathway. *Acta Pharmacologica Sinica*.

[76] Gao Y., Li J., Chu S. (2020). Ginsenoside Rg1 protects mice against streptozotocin-induced type 1 diabetic by modulating the NLRP3 and Keap1/Nrf2/HO-1 pathways. *European Journal of Pharmacology*.

[77] Li Q., Xiang Y., Chen Y., Tang Y., Zhang Y. (2018). Ginsenoside Rg1 protects cardiomyocytes against hypoxia/reoxygenation injury via activation of Nrf2/HO-1 signaling and inhibition of JNK. *Cellular Physiology and Biochemistry*.

[78] Gao Y., Chu S. F., Zhang Z. (2019). Ginsenoside Rg1 prevents acetaminophen-induced oxidative stress and apoptosisviaNrf2/ARE signaling pathway. *Journal of Asian Natural Products Research*.

[79] Dong C., Liu P., Wang H., Dong M., Li G., Li Y. (2019). Ginsenoside Rb1 attenuates diabetic retinopathy in streptozotocin-induced diabetic rats1. *Acta Cirúrgica Brasileira*.

[80] Jiang Y., Zhou Z., Meng Q. T. (2015). Ginsenoside Rb1 treatment attenuates pulmonary inflammatory cytokine release and tissue injury following intestinal ischemia reperfusion injury in mice. *Oxidative Medicine and Cellular Longevity*.

[81] Liu X., Gu X., Yu M. (2018). Effects of ginsenoside Rb1 on oxidative stress injury in rat spinal cords by regulating the eNOS/Nrf2/HO-1 signaling pathway. *Experimental and Therapeutic Medicine*.

[82] Xu H., Jiang Y., Yu K., Zhang X., Shi Y. (2022). Effect of ginsenoside Rh1 on proliferation, apoptosis, and oxidative stress in vascular endothelial cells by regulation of the nuclear erythroid 2-related factor-2/heme oxygenase-1 signaling pathway. *Journal of Cardiovascular Pharmacology*.

[83] Zhang Z., Yang K., Mao R. (2022). Ginsenoside Rg1 inhibits oxidative stress and inflammation in rats with spinal cord injury via Nrf2/HO-1 signaling pathway. *Neuroreport*.

[84] Mei X., Feng H., Shao B. (2020). Alleviation of sepsis-associated encephalopathy by ginsenoside via inhibition of oxidative stress and cell apoptosis: an experimental study. *Pakistan Journal of Pharmaceutical Sciences*.

[85] Wang X. M., She C., Li Q. (2020). Ginsenoside Rh3 activates Nrf2 signaling and protects endometrial cells from oxygen and glucose deprivation-reoxygenation. *Aging (Albany NY)*.

[86] Liu M., Bai X., Yu S. (2019). Ginsenoside re inhibits ROS/ASK-1 dependent mitochondrial apoptosis pathway and activation of Nrf2-antioxidant response in beta-amyloid-challenged SH-SY5Y cells. *Molecules*.

[87] Zeng X., Li J., Li Z. (2015). Ginsenoside Rd mitigates myocardial ischemia-reperfusion injury via Nrf2/HO-1 signaling pathway. *International Journal of Clinical and Experimental Medicine*.

[88] Yang Q., Lin J., Zhang H. (2019). Ginsenoside compound K regulates amyloid *β* via the Nrf2/Keap1 signaling pathway in mice with scopolamine hydrobromide-induced memory impairments. *Journal of Molecular Neuroscience*.

[89] Zhao Y., Wang Y., Zhang M., Gao Y., Yan Z. (2021). Protective effects of ginsenosides (20R)-Rg3 on H2O2-induced myocardial cell injury by activating Keap-1/Nrf2/HO-1 signaling pathway. *Chemistry & Biodiversity*.

[90] Chen S., Li X., Wang Y. (2019). Ginsenoside Rb1 attenuates intestinal ischemia/reperfusion‑induced inflammation and oxidative stress via activation of the PI3K/Akt/Nrf2 signaling pathway. *Molecular Medicine Reports*.

[91] Zhuang C. L., Mao X. Y., Liu S. (2014). Ginsenoside Rb1 improves postoperative fatigue syndrome by reducing skeletal muscle oxidative stress through activation of the PI3K/Akt/Nrf2 pathway in aged rats. *European Journal of Pharmacology*.

[92] Hwang Y. P., Jeong H. G. (2010). Ginsenoside Rb1 protects against 6-hydroxydopamine-induced oxidative stress by increasing heme oxygenase-1 expression through an estrogen receptor-related PI3K/Akt/Nrf2-dependent pathway in human dopaminergic cells. *Toxicology and Applied Pharmacology*.

[93] Wang X., Chen L., Wang T. (2015). Ginsenoside Rg3 antagonizes adriamycin-induced cardiotoxicity by improving endothelial dysfunction from oxidative stress _via_ upregulating the Nrf2-ARE pathway through the activation of akt. *Phytomedicine*.

[94] Xiong J., Yang J., Yan K., Guo J. (2021). Ginsenoside Rk1 protects human melanocytes from H2O2‑induced oxidative injury via regulation of the PI3K/AKT/Nrf2/HO‑1 pathway. *Molecular Medicine Reports*.

[95] Nan F., Sun G., Xie W. (2019). Ginsenoside Rb1 mitigates oxidative stress and apoptosis induced by methylglyoxal in SH-SY5Y cells via the PI3K/Akt pathway. *Molecular and Cellular Probes*.

[96] Li W., Wang J. Q., Zhou Y. D. (2020). Rare ginsenoside 20(R)-Rg3 inhibits D-galactose-induced liver and kidney injury by regulating oxidative stress-induced apoptosis. *The American Journal of Chinese Medicine*.

[97] Liu H., Chen W., Lu P., Ma Y., Liang X., Liu Y. (2021). Ginsenoside Rg1 attenuates the inflammation and oxidative stress induced by diabetic nephropathy through regulating the PI3K/AKT/FOXO3 pathway. *Ann Transl Med.*.

[98] Xie W., Zhou P., Qu M. (2020). Ginsenoside re attenuates high glucose-induced RF/6A injury via regulating PI3K/AKT inhibited HIF-1*α*/VEGF signaling pathway. *Frontiers in Pharmacology*.

[99] Chen L., Yao H., Chen X. (2018). Ginsenoside Rg1 decreases oxidative stress and down-regulates Akt/mTOR signalling to attenuate cognitive impairment in mice and senescence of neural stem cells induced by D-galactose. *Neurochemical Research*.

[100] Li J., Cai D., Yao X. (2016). Protective effect of ginsenoside Rg1 on hematopoietic stem/progenitor cells through attenuating oxidative stress and the Wnt/*β*-catenin signaling pathway in a mouse model of d-galactose-induced aging. *International Journal of Molecular Sciences*.

[101] Zu G., Guo J., Che N. (2016). Protective effects of ginsenoside Rg1 on intestinal ischemia/reperfusion injury-induced oxidative stress and apoptosis via activation of the Wnt/*β*-catenin pathway. *Scientific Reports*.

[102] Shao X., Chen C., Miao C. (2019). Expression analysis of microRNAs and their target genes during experimental diabetic renal lesions in rats administered with ginsenoside Rb1 and trigonelline. *Die Pharmazie*.

[103] Hagar H., Husain S., Fadda L. M., Attia N. M., Attia M. M. A., Ali H. M. (2019). Inhibition of NF-*κ*B and the oxidative stress -dependent caspase-3 apoptotic pathway by betaine supplementation attenuates hepatic injury mediated by cisplatin in rats. *Pharmacological Reports*.

[104] Ye Y., Shan Y., Bao C., Hu Y., Wang L. (2018). Ginsenoside Rg1 protects against hind-limb ischemia reperfusion induced lung injury via NF-*κ*B/COX-2 signaling pathway. *International Immunopharmacology*.

[105] Song W., Wei L., Du Y., Wang Y., Jiang S. (2018). Protective effect of ginsenoside metabolite compound K against diabetic nephropathy by inhibiting NLRP3 inflammasome activation and NF-*κ*B/p38 signaling pathway in high-fat diet/streptozotocin-induced diabetic mice. *International Immunopharmacology*.

[106] Hou J., Kim S. (2018). Possible role of ginsenoside Rb1 in skin wound healing via regulating senescent skin dermal fibroblast. *Biochemical and Biophysical Research Communications*.

[107] Chen J., Liu G. Z., Sun Q. (2019). Protective effects of ginsenoside Rg3 on TNF-*α*-induced human nucleus pulposus cells through inhibiting NF-*κ*B signaling pathway. *Life Sciences*.

[108] Li Y., Hou J. G., Liu Z. (2021). Alleviative effects of 20(R)-Rg3 on HFD/STZ-induced diabetic nephropathy via MAPK/NF-*κ*B signaling pathways in C57BL/6 mice. *Journal of Ethnopharmacology*.

[109] Hou J., Yun Y., Xue J., Jeon B., Kim S. (2020). Doxorubicin-induced normal breast epithelial cellular aging and its related breast cancer growth through mitochondrial autophagy and oxidative stress mitigated by ginsenoside Rh2. *Phytotherapy Research*.

[110] Ren B., Feng J., Yang N., Guo Y., Chen C., Qin Q. (2021). Ginsenoside Rg3 attenuates angiotensin II-induced myocardial hypertrophy through repressing NLRP3 inflammasome and oxidative stress via modulating SIRT1/NF-*κ*B pathway. *International Immunopharmacology*.

[111] Zhu Y., Zhu C., Yang H., Deng J., Fan D. (2020). Protective effect of ginsenoside Rg5 against kidney injury via inhibition of NLRP3 inflammasome activation and the MAPK signaling pathway in high-fat diet/streptozotocin-induced diabetic mice. *Pharmacological Research*.

[112] Zhou J., Zhang H. A., Lin Y. (2014). Protective effect of ginsenoside against acute renal failure via reduction of renal oxidative stress and enhanced expression of ChAT in the proximal convoluted tubule and ERK1/2 in the paraventricular nuclei. *Physiological Research*.

[113] Chen X. C., Zhou Y. C., Chen Y., Zhu Y. G., Fang F., Chen L. M. (2005). Ginsenoside Rg1 reduces MPTP-induced substantia nigra neuron loss by suppressing oxidative stress. *Acta Pharmacologica Sinica*.

[114] Zhou P., Lu S., Luo Y. (2017). Attenuation of TNF-*α*-induced inflammatory injury in endothelial cells by ginsenoside Rb1 via inhibiting NF-*κ*B, JNK and p38 signaling pathways. *Frontiers in Pharmacology*.

[115] Cong L., Chen W. (2016). Neuroprotective effect of ginsenoside Rd in spinal cord injury rats. *Basic & Clinical Pharmacology & Toxicology*.

[116] Zhang X., Wang L., Guo R. (2021). Ginsenoside Rb1 ameliorates diabetic arterial stiffening via AMPK pathway. *Frontiers in Pharmacology*.

[117] Saw C. L., Yang A. Y., Cheng D. C. (2012). Pharmacodynamics of ginsenosides: antioxidant activities, activation of Nrf2, and potential synergistic effects of combinations. *Chemical Research in Toxicology*.

[118] Du N., Xu Z., Gao M., Liu P., Sun B., Cao X. (2018). Combination of ginsenoside Rg1 and astragaloside IV reduces oxidative stress and inhibits TGF-&beta;1/Smads signaling cascade on renal fibrosis in rats with diabetic nephropathy. *Drug Design, Development and Therapy*.

